# The PI3K/AKT axis modulates AATF activity in Wilms’ tumor cells

**DOI:** 10.1002/2211-5463.12500

**Published:** 2018-09-04

**Authors:** Peng Jing, Jiaqiong Zou, Kegui Weng, Pei Peng

**Affiliations:** ^1^ Department of Pediatric Surgery Affiliated Hospital of Northern Sichuan Medical College Nanchong China; ^2^ Department of Clinical Medicine North Sichuan Medical College Nanchong China; ^3^ Department of Clinical Laboratory the First Affiliated Hospital of Chengdu Medical College Nanchong China; ^4^ Chongqing Cancer Institute Chongqing Cancer Hospital Chongqing University Cancer Hospital China; ^5^ Department of Clinical Laboratory the People's Hospital of Hanchuan/Hanchuan Hospital of People's Hospital Affiliated to Wuhan University China

**Keywords:** AATF, growth, invasion, migration, PI3K/AKT axis, Wilms’ tumor

## Abstract

Previous studies have reported excessive expression of apoptosis‐antagonizing transcription factor (AATF) in various tumors, where it reinforces the generation and development of cancers and is linked to the clinical outcome. Nevertheless, the expression and influence of AATF in Wilms’ tumor (WT) is largely unknown. Here, we discovered that AATF expression was markedly increased in WT tissues as compared to the surrounding normal tissues. Elevated levels of AATF expression were related to tumor relapse and pulmonary metastasis, congruent with it being a predictor of clinical outcome in people suffering from WT. Proliferation, invasion, and migration of WT cells were suppressed by knockdown of AATF and promoted by AATF overexpression *in vitro*. Furthermore, the tumor generation capability of WT cells noticeably decreased after knockout of AATF *in vivo*. The phosphoinositide‐3‐kinase (PI3K)/AKT pathway modulated the activity of AATF in WT. The findings of our study indicate that AATF expression is increased in WT and can serve as a predictor of clinical outcome; in addition, it may enhance the development of WT via the PI3K/AKT axis and may be a promising marker for WT diagnosis and therapy.

**Abbreviations**
AATF: apoptosis‐antagonizing transcription factor
MTS: 3‐(4,5‐dimethylthiazol‐2‐yl)‐5‐(3‐carboxymethoxyphenyl)‐2‐(4‐sulfophenyl)‐2*H*‐tetrazolium
PI3K: phosphoinositide‐3‐kinase
sh: short hairpin
TF: transcription factor
WT: Wilms’ tumor

Wilms’ tumor (WT) ranks as the fourth most prevalent cancer in children and the most prevalent type of kidney cancer in children 1. It contributes to 6–14% of tumors in children and 95% of all kidney cancers in children 1, 2. Despite the fact that multimodal treatment increases the overall cure rate, recurrence is present in almost 15% of patients suffering from favorable histology of WT, as well as in 50% of patients suffering from anaplastic WT 3, 4. The insufficient response to contemporary therapy requires the generation of innovative strategies for treating WT.

Transcription factors (TFs) such as apoptosis‐antagonizing transcription factor (AATF, also known as TRB), are specific to RNA polymerase II, indicating their modulation of cell death 5. At the same time, AATF plays a role in such processes as proliferation, stress reactions to DNA injury, and regulation of the cell cycle 6, 7. AATF is crucial in stress reactions related to DNA injury, such as the stimulation of p53 and, possibly, p21 5, 7, 8, 9. Excessive AATF expression is present in some human leukemic cells 10, 11. AATF blockage noticeably inhibits the growth of malignant tumors and increases sensitivity to chemotherapy in murine xenografts 12. These findings indicate that AATF can serve as an innovative target in terms of tumor treatment. Nevertheless, the current understanding of the role of AATF in WT is insufficient.

Our research reveals that AATF expression is elevated in WT in comparison with surrounding normal tissues. AATF overexpression is shown to activate the migration and invasion of malignant cells via the phosphoinositide‐3‐kinase (PI3K) /AKT axis in WT.

## Materials and methods

### Samples

Samples of WT along with the surrounding normal tissues were obtained from Hanchuan Hospital of People's Hospital affiliated to Wuhan University. Fifty‐six WT samples were acquired from 2012 to 2016; the samples were fixed in formalin and embedded in paraffin. Twenty fresh samples of WT along with the surrounding tissues were surgically obtained and refrigerated using liquid nitrogen. Informed consent was obtained from each subject, and the study methodologies have been approved by Hanchuan Hospital of People's Hospital affiliated to Wuhan University; the article is in accordance with the ARRIVE Guidelines for reporting *in vivo* animal experiments.

### Immunohistochemistry

In brief, after baking at 65 °C for 2 h, 5‐μm‐thickness sections were deparaffinized in xylene, hydrated using a graded series of alcohol (100%, 95%, and 85%) and rinsed with PBS. Antigenic retrieval was performed by immersing in citric acid and microwaving. To block any non‐specific binding, the sections were treated using 0.3% hydrogen peroxide solution for 15 min. The sections were then incubated overnight at 4 °C with AATF antibody (Sigma‐Aldrich, St Louis, MO, USA, 1 : 100) and examined using HRP EnVision Systems (Dako, Shanghai, China). Finally, sections were counterstained with hematoxylin and visualized.

### WT cell generation

Fresh malignant samples from a WT patient were used for constructing WT cell lines, as previously described 13. The samples were washed using Hanks’ solution containing penicillin and no calcium. The samples were cut into pieces and digested in a solution with 0.24% EDTA. Single cells were cultivated in flasks in DMEM (Thermo Fisher Scientific, Waltham, MA, USA) supplemented with 15% FBS (Thermo Fisher Scientific).

### Lentiviral transfection of WT cells

Insertion of short hairpin (sh) ‐AATF was carried out using the lentiviral vector pLL3.7. Infected lentiviruses were retrieved 48 h after transfection. Using the X‐tremeGENE HP DNA Transfection Reagent (Thermo Fisher Scientific), the AATF plasmids were transfected into WT cells.

### Real‐time RT‐PCR (qRT‐PCR)

Total RNA was isolated from WT samples. RNA from the surrounding tissue samples was extracted using TRIzol (Sigma‐Aldrich). The purified RNA was diluted using 30 μL RNase‐free water. Generation of cDNA was conducted on 2 μg of total RNA by using PrimeScript™ RT reagent kit (TaKaRa, Dalian, Liaoning, China). SYBR Premix Ex Taq II kit and the Applied Biosystems (Thermo Fisher Scientific) 7500 Quantitative PCR system were used for performing PCR. The expression of β‐actin was used for the normalization of the expression of target genes. Relative mRNA concentrations were evaluated according to *C*_t_ and normalized.

### Western blotting

The Wilms' tumor cells, stably transfected Wilms' tumor cells and 40 frozen specimens were obtained for protein separation purposes. Proteins were separated and quantified. The proteins were isolated using SDS/PAGE and transferred to nitrocellulose filter membranes. Signals were evaluated using a chemiluminescence imaging system after incubation with secondary antibodies conjugated with horseradish peroxidase.

### Apoptosis assays

Apoptosis was analyzed by nuclear staining with Hoechst 33258 (Invitrogen, Carlsbad, CA, USA). Cells were seeded in 12‐well plates (1 × 10^5^ cells·mL^−1^). PBS was used to wash the plates three times after cultivating for 48 h. Hoechst 33342 solution (500 μL) was added to every well before 30 min incubation in the dark at 37 °C. A fluorescence microscope (Olympus, Tokyo, Japan) was used to evaluate nuclear DNA staining. One hundred cells were counted at random from 10 visual fields. Proportions of cells with fluorescence staining were presented in the form of the ratio of dead cells/all calculated cells.

### MTS assay

A 3‐(4,5‐dimethylthiazol‐2‐yl)‐5‐(3‐carboxymethoxyphenyl)‐2‐(4‐sulfophenyl)‐2*H*‐tetrazolium (MTS) assay was performed as previously reported 14. Briefly, cells from different groups were cultivated in 96‐well plates at 2000 cells/well. A MTS assay kit (Promega, Madison, WI, USA) was used. Every assay was carried out in triplicate. The procedures were conducted three times.

### Wound‐healing assay

Wilms’ tumor cells from distinct groups were cultivated in 96‐well plates and were scraped using a 100‐μL pipette tip at 70% confluence to generate two parallel wounds. The cells were washed with PBS and incubated for 24 h in the medium without serum, at 37 °C. A Leica DMI4000B microscope (Leica, Wetzlar, Germany) was used for photographing the cells every 8 h.

### Transwell assay

Matrigel™ (BD Biosciences, San Jose, CA, USA) was diluted to 1 : 7 using the basal medium without serum. Fifty microliters of Matrigel Matrix solution was added into each chamber (Corning, Lowell, MA, USA). One hundred microliters of the suspension of WT cells (2 × 10^5^ cells·mL^−1^) from different groups was seeded into the chambers and incubated in the basal medium without serum. Five hundred microliters of medium containing 10% FBS was added to the chambers at the bottom. After 24 h, the cells were removed from the top chambers using cotton swabs. PBS was utilized to wash the inserts three times. Cells that moved below were fixed with paraformaldehyde (4%) and stained with crystal violet (1%).

### Clone formation assay

Wilms’ tumor cells were seeded into six‐well plates at the density of 1000 cells/well. Cells were cultivated for 2 weeks and subsequently fixed using 4% paraformaldehyde. The plates were subsequently seasoned, and the clones were quantified.

### Animal models

To construct subcutaneous malignancy models, male nude BALB/C mice aged 5–6 weeks were randomized into four groups: sh‐control, vector, sh‐AATF, vector and AATF. The mice received a subcutaneous injection of 100 μL of a solution containing 2 × 10^6^ WT cells. The tumor growth was documented every other day. Immunohistochemical staining was applied for evaluating AATF expression.

### Statistical analysis

The chi‐square test and ANOVA were utilized in order to evaluate the relationship between the clinicopathology and expression of AATF. Multivariate and univariate evaluations of predictors of clinical outcome were carried out using Cox's proportional hazards model. Data were regarded as significant with two‐tailed *P* < 0.05. spss 13.0 software (SPSS Inc., Chicago, IL, USA) was used for data evaluation.

## Results

### Increased AATF expression in WT in comparison to surrounding tissues

Immunohistochemistry, western blotting, and qRT‐PCR were carried out on samples of WT and surrounding tissues in order to evaluate the expression of AATF. qRT‐PCR results showed that AATF expression was noticeably increased in WT samples in comparison with that in surrounding tissues, and the difference between these two groups was statistically significant (Fig. 1A, *P *< 0.05). Five paired specimens were randomly selected to evaluate AATF translation by western blotting. The protein level of AATF was enhanced in WT (Fig. 1B). The above findings were verified using immunohistochemistry: AATF expression was increased in malignant samples compared with that in normal samples (Fig. 1C). Furthermore, the influence of AATF expression on the clinical outcome of patients suffering from WT was examined using univariate Cox's regression analysis (Table 1). We next analyzed the level of AATF and clinicopathological features. Our results demonstrated that AATF expression was positively correlated with tumor recurrence or lung metastasis (Table 2). These results revealed that AATF is increased in WT in comparison to surrounding tissues.

**Figure 1:** Expression of AATF in human WT. (A) Real‐time RT‐PCR analysis of *AATF* mRNA levels in WT tissues (Tumor) and adjacent normal tissues (Normal). *P < 0.05 (Student's *t* test). (B) AATF protein levels in WT tissues and adjacent normal tissues were analyzed by western blotting. (C) Immunohistochemical staining of AATF in non‐tumor and primary WT tissues.

**Table 1:** Apoptosis‐antagonizing transcription factor expression in WT and adjacent non‐cancer tissues

	AATF expression		*P*
	High	Low	
WT	38	18	<0.05
Adjacent non‐cancer samples	23	33	

**Table 2:** The relationship between AATF expression and clinicopathological features

Clinicopathological characteristic	AATF expression		*P*
	High	Low	
Gender			
Male	18	10	0.12
Female	20	8	
Lung metastasis/recurrence			
Yes	25	3	0.0065
No	13	15	
Tumor size			
<8 cm	17	11	0.034
≥8 cm	21	7	

### AATF‐stimulated WT cell proliferation

We constructed WT cell lines from fresh malignant samples from a person suffering from WT to evaluate the influence of AATF on the development of WT cells. Knockdown was subsequently carried out using lentiviral sh‐AATF. The efficiency of the above procedures is presented in Fig. 2A. A MTS assay was applied for quantifying cell survival. The results showed that knockdown of AATF markedly suppressed WT cell proliferation (Fig. 2B,C; *P *< 0.05). Moreover, the number of sh‐AATF cell clones was noticeably lower than in the control group, and the difference between these two groups was statistically significant (Fig. 2D; *P *< 0.05). In addition, overexpression AATF promoted WT cell proliferation (Fig. 2E–G). Overexpression of AATF blocked doxorubicin‐induced apoptosis in WT cells (Fig. 2H,I). These findings indicate that AATF expression could promote the proliferation of WT cells.

**Figure 2:** Effects of AATF on the proliferation of WT cells. (A) AATF expression was analyzed by western blotting after sh‐AATF transfection. (B) Cell viability was analyzed by MTS assay at different time points. Data are expressed as mean ± SD from three experiments; *P < 0.05 (ANOVA). (C) Cell number was analyzed at different time points. Data are expressed as mean ± SD from three experiments; *P < 0.05 (ANOVA). (D) Effects of AATF on colony formation. Data are expressed as mean ± SD from three experiments; *P < 0.05 (Student's *t* test). (E) WT cells were transfected with AATF for 24 h, AATF expression was analyzed by western blotting. (F) WT cells were transfected with AATF for 24 h, cell viability was analyzed by MTS assay at different time points. Data are expressed as mean ± SD from three experiments, *P < 0.05 (ANOVA). (G) WT cells were transfected with AATF for 24 h, and cell number was analyzed at different time points. Data are expressed as mean ± SD from three experiments; *P < 0.05 (ANOVA). (H) WT cells were transfected with AATF for 24 h, cells were treated with 1 μm doxorubicin for another 24 h, and apoptosis was analyzed by nuclear staining. Data are expressed as mean ± SD from three experiments; *P < 0.05. (I) WT cells were transfected with AATF for 24 h, cells were treated with 1 μm doxorubicin (Dox) for another 24 h, and cleaved caspase 3 was detected by western blotting.

### AATF enhanced the migration of WT cells

Considering that AATF expression was able to affect WT metastasis, a Transwell assay and wound‐healing assay were utilized to verify the correlation between AATF expression and cell invasion and migration *in vitro*. The stable AATF reduction increased the healing distances of control cells (Fig. 3A). Invasion through pores was limited in the sh‐AATF group in comparison with that in the control, as shown in Fig. 3B. The differences in the wounding healing and invasion cells are statistically significant (*P < 0.05). These findings demonstrate that suppressed expression of AATF inhibits the invasion and migration capability of WT cells.

**Figure 3:** Effects of AATF on migration and invasion of WT cells. (A) WT cells were transfected with sh‐AATF, and the migratory behavior was analyzed using the wound‐healing assay. Data are expressed as mean ± SD from three experiments; *P < 0.05 (Student's *t* test). (B) WT cells were transfected with sh‐AATF, and their invasiveness was analyzed using Transwell assays. Data are expressed as mean ± SD from three experiments; *P < 0.05 (Student's *t* test).

### AATF affects the PI3K/AKT axis in WT

Previous studies have shown that AATF participates in signaling pathways such as the PI3K/AKT pathway 6. Western blotting was carried out to examine the pathways involved in WT. As a result of AATF knockdown, total and phosphorylated AKT were suppressed (Fig. 4A). Exogenous AATF expression increased the levels of total and phosphorylated AKT (Fig. 4B), which was inhibited by the AKT inhibitor perifosine, indicating that AATF is implicated in WT via the PI3K/AKT pathway, as well as via downstream translation.

**Figure 4:** Apoptosis‐antagonizing transcription factor affects AKT signaling in WT cells. (A) WT cells were transfected with sh‐con or sh‐AATF; the indicated protein levels were analyzed by western blotting. (B) WT cells were transfected with a vector or AATF. The indicated protein level was analyzed by western blotting.

### The PI3K/AKT axis may modulate AATF activity in WT cells

WT cells overexpressing AATF were treated with perifosine, a PI3K/AKT signaling pathway inhibitor. It was found that proliferation of the cells was markedly inhibited after perifosine treatment (Fig. 5A,B). Moreover, findings of Transwell assays show that blocking PI3K/AKT noticeably suppressed the invasion stimulated by AATF (Fig. 5C). In addition, perifosine inhibited proliferation of sh‐con cells, but had no effects on sh‐AATF cells (Fig. 5D,E). The above data indicated that the PI3K/AKT signaling pathway at least partly modulates AATF activity in WT cells.

**Figure 5:** AKT signaling affects AATF functions in WT cells. Effects of perifosine on AATF‐enhanced cell proliferation (A), cell number (B) and invasion (C), and effects of perifosine on sh‐AATF cell proliferation (D) and cell number (E). Data in (A,B) are expressed as mean ± SD from three experiments; *P < 0.05 (ANOVA). Data in (C) are expressed as mean ± SD from three experiments; *P < 0.05 (Student's *t* test).

### AATF‐enhanced tumor development

To verify the influence of AATF on tumor development, subcutaneous xenografts were constructed in nude mice. The tumor volume in the sh‐AATF group was lower than in the shRNA‐negative control (shRNA‐NC) group 20 days after inoculation. The tumor size in the AATF group was greater than in the control group. No difference was observed in tumor size between the shRNA‐NC and vehicle groups (Fig. 6A). The tumor weight was lower in the sh‐AATF group than in the shRNA‐NC group. It was enhanced in the AATF group, and no difference was observed between the control and shRNA‐NC groups (Fig. 6B). By immunohistochemistry and Ki‐67 staining, it was demonstrated that AATF knockdown markedly suppressed the proliferation of tumor cells, that is, that tumor cell proliferation was enhanced by AATF (Fig. 6C). Western blotting results showed that AKT activation decreased in sh‐AATF group in comparison with the shRNA‐NC group, but increased in the AATF group relative to the vector group (Fig. 6D).

**Figure 6:** AATF enhanced tumor growth *in vivo*. (A) Tumor volume in each group. *n *= 6 in each group; for indicated comparisons, *P < 0.05 (ANOVA). (B) Tumor weight in each group. *n *= 6 in each group; for indicated comparisons, *P < 0.05 (ANOVA). (C) Expression of Ki‐67 (cell proliferation marker) in xenograft tumors analyzed by immunohistochemical staining. (D) Western blotting of p‐AKT in each group.

## Discussion

As the most prevalent kidney tumor in children, WT has a prevalence rate of 1 : 10 000 among children 15, 16. The clinical outcome of WT relies on various factors such as age, cancer stage, size of malignancy before surgery, and histology 16, 17. Determining the molecular factors related to the clinical outcome of WT is crucial.

AATF has been discovered in recent years by different groups 5, 18. It has been found that AATF participates in the regulation of cell death and transcription 6, 12, 19. AATF participates in tumor progression and proliferation because of its contribution to growth and viability in various tumors 20, 21, 22, 23. Our study explored the expression and activity of AATF in WT. The results showed that increased AATF expression was linked to tumor relapse and pulmonary metastasis in WT patients. We also showed that patients with increased expression of AATF had lower survival rates. Furthermore, increased expression of AATF served as an independent risk factor. Nevertheless, the understanding of the contribution of AATF to WT progression is still insufficient. We found that increased expression of AATF enhanced the proliferation, invasion, and migration of WT cells. It also promoted the ability of WT cells to generate tumors *in vivo*. Consequently, AATF is able to participate in the development of WT through various mechanisms.

It is widely accepted that the PI3K/AKT axis participates in protein generation, proliferation, and viability of malignant cells, thus serving as a crucial downstream pathway of AATF 24, 25. As a result, AATF participates in the migration, proliferation, and invasion of WT cells, possibly via the PI3K/AKT axis.

## Conclusion

In conclusion, our research showed increased AATF expression in WT and the relationship between it and the clinical outcome of patients suffering from WT. Increased expression of AATF is a predictor of the clinical outcome of WT. AATF enhanced the invasion, proliferation, and migration of WT cells. Moreover, AATF reinforced the generation of malignant cells in WT possibly via the PI3K/AKT axis.

## Author contributions

In this work, PJ and PP conceived the study and designed the experiments. JZ and KW contributed to the data collection, performed the data analysis, and interpreted the results. PJ wrote the manuscript. PP contributed to the critical revision of the article. All authors read and approved the final manuscript.
